# Psychometric properties of the self-report version of the strengths and difficulties questionnaire in the Ecuadorian context: an evaluation of four models

**DOI:** 10.1186/s40359-019-0328-6

**Published:** 2019-08-06

**Authors:** Paúl Arias-Medina

**Affiliations:** Faculty of Psychology, University of Cuenca, Cuenca, Ecuador

**Keywords:** Mental health, Children, Psychometrics, Validity, Reliability, SDQ

## Abstract

**Background:**

This study evaluates the psychometric properties of four models of the Strengths and Difficulties Questionnaire (SDQ) in a sample of 1470 children and adolescents from Biblián, Ecuador. The instrument has been used by researchers and students. However, there are not reports that show that the instrument is valid or reliable in the Ecuadorian context.

**Methods:**

Reliability was evaluated through Cronbach’s Alpha, McDonald’s Omega, Intra-class Correlations and Greatest Lower Bound (GLB). Exploratory Factor Analysis (EFA) and Confirmatory Factor Analysis (CFA) with polychoric correlation matrix and Diagonally Weighted Least Square (DWLS) estimator is performed in each model. Due to possible readability problems, CFA was performed in three age groups. Measurement invariance analysis across biological sex and two groups of age is carried out.

**Results:**

CFA and reliability analysis revealed poor construct validity of the original version of SDQ. Three additional factor structures were tested. A version that includes a prosocial subscale, and ҅ internalizing ҆ subscale and an ҅ externalizing ҆ subscale has the best yet insufficient construct validity properties among the four models (CFI = .858, TLI *=* .844, RMSEA *=* .055, WRMR *=* 1.588). Cronbach’s Alpha for the subscales ranged from .44 to .71, McDonald’s Omega from .22 to .606, GLB from .612 to .693, and ICC from .385 to .63. Measurement invariance analysis found no evidence of invariance across sex groups and evidence of partial invariance across age groups.

**Conclusions:**

The four tested models have questionable psychometric properties. Consequently, the use of the SDQ in the Ecuadorian context is not advisable. The three-factor first-order model of the SDQ that shows the best validity and reliability properties does not have undisputed psychometric properties. Comparisons across groups of age and/or sex using the SDQ should not be made.

## Background

International migration is prevalent in Biblián, Ecuador. In the last years, a number of projects have studied the effects of international migration on monetary and non-monetary dimensions. Particular attention is directed towards children and adolescents since they are considered a vulnerable group and a global estimated of 13.4% of them are affected by any mental disorder [2]. The SDQ, henceforth SDQ, [1, 3] is a widely popular screening tool for psychosocial problems and strengths. The questionnaire was developed as a behavioural screening scale of 25 items that includes an impact supplement that inquires about distress, social impairment, burden and chronicity in a brief manner that does not require much time to respond. There are two additional questionnaires aimed at parents and teachers with slight modifications. The SDQ has also been used to monitor the effectiveness of routine clinical services or as a measure of child well-being in community settings such as schools. The scale also distinguishes between clinic and community samples and its popularity relies on the fact that it can be used for screening, clinical assessment, treatment-outcome measure, and as a research tool [4]. Despite the self-respondent version was designed to be answered by children and adolescents ages 11 to 17 years old, other research has validated the SDQ in children as young as 6 years old [5–7]. However, other investigation has also shown that the readability of the questionnaire is deficient in children under 13 years old [8].

The instrument has been widely used around the world in countries like Brazil [9, 10], England [5, 11, 12], Australia [13–15], Bangladesh [11, 16], United States of America [17], Finland [18], Belgium [19], Spain [20, 21], Italy [22], Greece [23], Gaza strip [24], China [25], among others [26, 27]. To the best of my knowledge, there is not any study of the psychometric properties of the SDQ in the Ecuadorian context. This paper reports the psychometric properties of the self-responded version of the SDQ to find out whether cultural and idiomatic characteristics of Ecuador affect its validity and reliability. Therefore, another factor structure might be more suitable for the Ecuadorian context, considering that the SDQ is rooted in Western psychological assessment [1]. This paper aims to evaluate different factor structures of the self-respondent version of the SDQ as part of an International Migration Project that aims to evaluate the non-monetary effects of migration.

## Method

### Participants

The original sample included 2129 observations, but 389 were deleted due to missing values in the questions of the SDQ. As for inclusion criteria, respondents had to be enrolled in school, and to be older than 4 and younger than 17 years old. The final set includes students from 7 to 17 years old (*M =* 12.77, *SD =* 2.42) from nine schools and high schools who completed all the questions of the SDQ (*n =* 1470). The schools are located in Biblián, Ecuador and its surrounding areas. Biblián is an Andean Ecuadorian town with a high migration prevalence. The information was collected from May to July 2015. The sample is composed of 740 boys and 730 girls. The data was collected in the PEACH (Problems, Expectations and Aspirations of Children) Survey of the VLIR-IUC Migration and Local Development Project.

### Instruments

The SDQ in its original version consists of 25 questions that include difficulties measured as emotional symptoms (5 items), conduct problems (5 items), hyperactivity/inattention (5 items) and peer relationship problems (5 items). Strengths are measured by a prosocial behaviour subscale (5 times), on a 3-point ordinal Likert scale (0: “not true”; 1 “somewhat true”; 2 “certainly true”). As stated before, the original five-factor structure is tested along with three other different configurations.

A sociodemographic questionnaire was applied along with the SDQ. Age group and biological sex are used for measurement invariance analysis.

### Procedure

The original Spanish translation was slightly modified to make it more comprehensible for Ecuadorian children by three professionals (a psychologist, an anthropologist and an educator). A pilot test was applied to a group of 52 children to guarantee a proper understanding of the questionnaire. As a result, some slight modifications were done to the Spanish version. The word “hiperactivo/a” (hyperactive) was eliminated in item 2 because it was not well understood; “Suelo tener” (I use to have) was replaced by “Frecuentemente tengo” (I frequently have) in item 3; “enfado” (get angry) was replaced by the synonym “enojo” in item 4; “gente” (people) was replaced by “compañeros” (mates/classmates) in item 5 and 14; “A menudo” (Oftentimes) was replaced by the synonym “Muchas veces” (Many times) in items 8, 13 and 20; “enfermo, lastimado o herido” (sick, hurt, or injured) was replaced by “lastimado o enfermo” (injured or sick) in item 9; “me muevo demasiado” (I move too much) was eliminated in item 10; “otros” (others) was replaced by “compañeros” (mates/classmates) and “manipulo” (manipulate) was replaced by “intimido” (intimidate) in item 12; “fácilmente pierdo la confianza en mí mismo/a” was eliminated of item 16; “niño/as más pequeño/as” (younger children) was replaced by “chicos (as) de menor edad que la mía” with the same meaning in item 17; item 19 was changed to “otros chicos (as) de mi edad me agreden o se burlan de mí” (other kids of my age assault or make fun of me) instead of “se meten conmigo” which was confusing for some kids; “Cojo” (take) was replaced by the synonym “Tomo” in item 22.

### Application

The SDQ was completed along with an extensive questionnaire as part of the PEACH (Problems, Expectations and Aspirations of Children) survey of the VLIR-IUC Migration and Local Development Project. Children and adolescents voluntarily answered the survey after obtaining written permission from their parents or main caregivers. Permission was granted by the authorities of the nine schools located in Biblián, Ecuador. The questionnaires and results guarantee confidentiality and anonymity of the participants.

### Data analysis

This paper evaluates four models suggested in other investigations around the world. First, the original five-factor first-order model, henceforth Model A [4, 17, 23, 28, 29]. This model includes a subscale of emotional symptoms (items 3, 8, 13, 16, 9), peer problems (items 6, 11, 14, 19, 23), conduct problems (items 5, 7, 12, 18, 22), hyperactivity/inattention problems (items 2, 10, 15, 21, 24) and prosocial behaviour (items 1, 4, 17, 20, 25). Second, a three-factor first-order model, henceforth Model B, that combines the emotional and peer subscales into a ‘internalizing’ subscale (items 3, 8, 13, 16, 9, 6, 11, 14, 19, 23), a behavioral subscale (items 5, 7, 12, 18, 22, 2, 10, 15, 21, 24), and a prosocial subscale (items 1, 4, 17, 20, 25) as proposed by Goodman & Goodman [12, 30]. Third, a second version of a three-factor first-order model, henceforth Model C, that includes an ‘internalizing’ subscale (items 3, 6, 8, 14, 16, 19, 23, 24), an ‘externalizing’ subscale (2, 5, 10, 12, 15, 18, 21, 22, 25) and a prosocial subscale (items 1, 4, 7, 9, 11, 14, 17, 20) [18, 19, 22]. Finally, a five-factor second-order model, henceforth model D, with the same first-order dimensions and items than the original version, but with an ‘internalizing’ and ‘externalizing’ second-order factors. The difference among models B and C is in the items that are included in each subscale (Fig. 1).

**Fig. 1:** Original and Alternative Factor Structures of the Strength and Difficulties Questionnaire

A descriptive analysis is carried out in order to analyse the distribution of the SDQ items.

Cronbach’s alpha, McDonald’s omega, Intra-class correlation coefficient, and Greatest Lower Bound were computed to assess the reliability of the complete questionnaire and its subscales [31–33]. Additionally, inter-item correlations and item-total correlations are computed.

The factorability of the matrix is determined by Bartlett’s sphericity test, Kaiser-Meyer-Olkin criteria and Henze-Zirkler test.

In order to perform EFA and CFA, the sample was randomly split into two subsamples (*n =* 735 each one).

Exploratory Factor Analysis (EFA) was used to determine the number of factors to be extracted following the Kaiser criterion [34]. Consequently, the components with Eigenvalues higher than 1.0 are retained. EFA is performed in the first subsample (*n =* 735).

Confirmatory Factor Analysis (CFA) with polychoric correlation matrix is used because of its adequacy to ordinal and non-normal data [35–38] with Diagonally Weighted Least Square (DWLS) estimator. The CFA was performed in the second subsample (*n =* 735). Additionally, in order to evaluate possible readability problems, all four models were tested in three age groups: First, the whole sample of children with ages ranging from 7 to 17 years old. Second, children from 7 to 12 years old. Third, children from 13 to 17 years old.

To assess goodness of fit, many indexes were used which cutoffs are the result of simulation studies [39–42]: Comparative Fit Index (CFI), Tucker-Lewis Index (TLI), Root-Mean-Square Error of Approximation (RMSEA) and Weighted Root-Mean-square Residual (WRMR). A model has a good fit if CFI ≥ .96, TLI ≥ .95 and RMSEA ≤ .05. CFI and TLI ≥ .90, RMSEA < .08 reflect acceptable fit and mediocre fit if .08 ≤ RMSEA ≤ .10, with CFI and TLI ≥ .9. When CFI or TLI < .90, or RMSEA > .10 the model should be rejected. Additionally, Weighted Root-Mean-Square Residual should be less than or equal to 1.00.

Measurement invariance was tested across age and sex groups for the model with the best goodness of fit and reliability indexes using the whole sample *(n =* 1470). Constraints were subsequently added in order to assess configural invariance, metric invariance, scalar invariance, and latent means invariance.

Statistical analysis was done using with R software 3.3.2 and lavaan package [43].

## Results

### Descriptive statistics

Main descriptive statistics are presented in Table 1. Given the categorical nature of the variables, it is recommended the use of polychoric correlation matrixes instead of Pearson correlations along with a Diagonally Weighted Least Squares estimator [35–38].

**Table 1:** Descriptive Statistics of the SDQ items

Item	Mean	Standard Deviation	median	skewness	Kurtosis
consid	2.61	.58	3	−1.19	.39
restles	1.67	.68	2	.53	−.78
somatic	1.41	.67	1	1.35	.45
shares	2.6	.59	3	−1.17	.35
tantrum	1.63	.76	1	.74	−.91
loner	1.37	.68	1	1.55	.9
obeys	2.33	.59	2	−.23	−.66
worries	2.02	.74	2	−.03	−1.2
caring	2.51	.63	3	−.9	−.24
fidgety	1.85	.78	2	.28	−1.3
friend	2.81	.49	3	−2.64	6.05
fights	1.36	.6	1	1.44	.99
unhappy	1.75	.78	2	.46	−1.22
popular	2.5	.63	3	−.87	−.29
distrac	1.82	.77	2	.33	−1.26
clingy	2.25	.76	2	−.46	−1.13
kind	2.68	.58	3	−1.6	1.52
lies	1.37	.62	1	1.43	.88
bullied	1.46	.72	1	1.22	−.01
helpout	2.46	.61	3	−.65	−.53
reflect	2.58	.6	3	−1.13	.24
steals	1.15	.45	1	3.08	8.65
oldbest	1.95	.79	2	.09	−1.39
afraid	1.68	.77	1	.62	−1.07
attends	2.35	.62	2	−.41	−.67

Item analysis results are presented in Table 2 along with item-total correlation coefficients including item-whole correlation, item-total standardized correlation, Item whole correlation corrected for item overlap and scale reliability, and item-whole correlation for the item against the scale without the item.

**Table 2:** Item analysis of the SDQ

Item	Item-total correlation	Item-total standardized correlation	Item whole correlation corrected for item overlap and scale reliability	Item whole correlation for this item against the scale without this item
consid	.3	.33	.27	.208
restles	.39	.37	.33	.285
somatic	.34	.32	.26	.236
shares	.2	.23	.16	.105
tantrum	.44	.41	.37	.332
loner	.36	.35	.3	.256
obeys	.42	.44	.41	.337
worries	.4	.36	.32	.29
caring	.29	.32	.26	.191
fidgety	.4	.37	.33	.283
friend	.24	.29	.22	.163
fights	.44	.44	.4	.353
unhappy	.5	.46	.44	.392
popular	.33	.36	.3	.238
distrac	.48	.45	.42	.373
clingy	.33	.29	.23	.213
kind-	.35	.39	.34	.266
lies	.39	.4	.36	.297
bullied	.45	.43	.39	.349
helpout	.19	.23	.16	.095
reflect-	.37	.4	.36	.285
steals	.37	.41	.36	.307
oldbest	.27	.24	.17	.149
afraid	.42	.38	.34	.307
attends	.46	.48	.46	.371

### Exploratory factor analysis

Factorability of the data was possible according to Bartlett’s sphericity test (χ^2^ = 2207.391, *df = 3*00, *p <* .01), Kaiser-Meyer-Olkin [44] measure of sampling adequacy (.804) and Henze-Zirkler multivariate normality test (*p < .*01).

Exploratory factor analysis results presented in Table 3 show that six factors with eigenvalues ranging from 1.103 to 3.648 should be retained and analysed that explain 43.16% of the variance (Fig. 2). It is also notable that there are some dimensions that have eigenvalues close to one.

**Table 3:** Eigenvalues and explained variance of the SDQ

Dimension	Eigenvalue	Explained variance	Cumulative variance
Dim.1	3.648	14.593	14.593
Dim.2	2.402	9.608	24.200
Dim.3	1.372	5.490	29.690
Dim.4	1.136	4.544	34.234
Dim.5	1.129	4.515	38.750
Dim.6	1.103	4.410	43.160
Dim.7	.993	3.972	47.132
Dim.8	.982	3.927	51.059
Dim.9	.947	3.786	54.845
Dim.10	.889	3.557	58.402
Dim.11	.874	3.496	61.897
Dim.12	.855	3.420	65.318
Dim.13	.835	3.342	68.659
Dim.14	.772	3.090	71.749
Dim.15	.751	3.005	74.754
Dim.16	.740	2.962	77.716
Dim.17	.697	2.788	85.03
Dim.18	.689	2.756	83.259
Dim.19	.677	2.708	85.967
Dim.20	.658	2.631	88.598
Dim.21	.619	2.475	91.072
Dim.22	.606	2.424	93.496
Dim.23	.576	2.305	95.802
Dim.24	.537	2.148	97.950
Dim.25	.513	2.050	100.000

**Fig. 2:** Number of extracted dimensions and its explained variance

### Confirmatory factor analysis and reliability

Confirmatory factor analysis performed in the four models led to factor loadings presented in Tables 4, 5, 6, and 7. Cronbach’s alpha, McDonald’s omega, intra-class correlation and GLB for each subscale are presented in the same tables.

**Table 4:** Factor loadings and internal consistency of Model A

	Age 7–17					Age 7–12					Age 13–17				
Item	ES	H	PP	CP	PB	ES	H	PP	CP	PB	ES	H	PP	CP	PB
somatic	.46	0	0	0	0	.39	0	0	0	0	.52	0	0	0	0
worries	.64	0	0	0	0	.56	0	0	0	0	.57	0	0	0	0
unhappy	.76	0	0	0	0	.73	0	0	0	0	.77	0	0	0	0
clingy	.41	0	0	0	0	.36	0	0	0	0	.47	0	0	0	0
afraid	.58	0	0	0	0	.62	0	0	0	0	.56	0	0	0	0
restles	0	.50	0	0	0	0	.43	0	0	0	0	.53	0	0	0
fidgety	0	.44	0	0	0	0	.46	0	0	0	0	.45	0	0	0
distrac	0	.52	0	0	0	0	.53	0	0	0	0	.52	0	0	0
reflect	0	−.46	0	0	0	0	−.41	0	0	0	0	−.55	0	0	0
attends	0	−.59	0	0	0	0	−.54	0	0	0	0	−.61	0	0	0
loner	0	0	.40	0	0	0	0	.39	0	0	0	0	.44	0	0
friend	0	0	−.30	0	0	0	0	−.32	0	0	0	0	−.30	0	0
popular	0	0	−.42	0	0	0	0	−.37	0	0	0	0	−.40	0	0
bullied	0	0	.61	0	0	0	0	.63	0	0	0	0	.50	0	0
oldbest	0	0	.18	0	0	0	0	.20	0	0	0	0	.24	0	0
tantrum	0	0	0	.38	0	0	0	0	.45	0	0	0	0	.43	0
obeys	0	0	0	−.53	0	0	0	0	−.44	0	0	0	0	−.57	0
figñhts	0	0	0	.48	0	0	0	0	.47	0	0	0	0	.57	0
lies	0	0	0	.43	0	0	0	0	.38	0	0	0	0	.53	0
steals	0	0	0	.49	0	0	0	0	.52	0	0	0	0	.60	0
consid	0	0	0	0	.53	0	0	0	0	.49	0	0	0	0	.48
shares	0	0	0	0	.41	0	0	0	0	.25	0	0	0	0	.51
caring	0	0	0	0	.48	0	0	0	0	.49	0	0	0	0	.55
kind	0	0	0	0	.67	0	0	0	0	.65	0	0	0	0	.63
helpout	0	0	0	0	.38	0	0	0	0	.33	0	0	0	0	.47
α	.70	.17	.18	.22	.62	.66	.16	.17	.23	.57	.71	.07	.04	.34	.65
ω	.62	.12	.05	.22	.52	.58	.15	.08	.25	.47	.61	.11	.04	.32	.55
ICC	.58	.14	.15	.25	.50	.57	.18	.15	.15	.42	.62	.11	.08	.26	.53
GLB	.67	.38	.29	.44	.54	.66	.37	.31	.38	.45	.71	.45	.27	.50	.57

*ES* Emotional Symptoms, *H* Hyperactivity, *PP* Peer Problems, *CP* Conduct Problems, *PB* Prosocial Behaviour, *α* Cronbach’s Alpha, *ω* McDonald’s Omega, *ICC* Intra-class correlation coefficient, *GLB* Greatest Lower Bound

**Table 5:** Factor loadings and internal consistency of Model B

	Age 7–17			Age 7–12			Age 13–17		
Item	IP	CP	PB	IP	CP	PB	IP	CP	PB
somatic	.44	0	0	.36	0	0	.49	0	0
worries	.61	0	0	.52	0	0	.53	0	0
unhappy	.70	0	0	.68	0	0	.70	0	0
clingy	.38	0	0	.34	0	0	.44	0	0
afraid	.55	0	0	.58	0	0	.52	0	0
loner	.37	0	0	.40	0	0	.44	0	0
friend	−.21	0	0	−.26	0	0	−.19	0	0
popular	−.33	0	0	−.33	0	0	−.32	0	0
bullied	.63	0	0	.65	0	0	.54	0	0
oldbest	.22	0	0	.22	0	0	.30	0	0
tantrum	0	.41	0	0	.49	0	0	.45	0
obeys	0	−.54	0	0	−.46	0	0	−.57	0
fights	0	.50	0	0	.50	0	0	.56	0
lies	0	.45	0	0	.41	0	0	.53	0
steals	0	.51	0	0	.55	0	0	.59	0
restles	0	.49	0	0	.42	0	0	.51	0
fidgety	0	.44	0	0	.46	0	0	.43	0
distrac	0	.51	0	0	.52	0	0	.51	0
reflect	0	−.44	0	0	−.40	0	0	−.52	0
attends	0	−.57	0	0	−.53	0	0	−.58	0
consid	0	0	.53	0	0	.51	0	0	.46
shares	0	0	.40	0	0	.24	0	0	.48
caring	0	0	.49	0	0	.48	0	0	.56
kind	0	0	.67	0	0	.64	0	0	.64
helpout	0	0	.38	0	0	.31	0	0	.49
α	.60	.34	.62	.59	.30	.57	.60	.37	.65
ω	.45	.23	.52	.42	.25	.46	.45	.27	.56
ICC	.57	.31	.50	.54	.29	.42	.55	.33	.53
GLB	.66	.53	.54	.60	.49	.45	.66	.59	.57

*IP* Internalizing Problems, *CP* Conduct Problems, *PB* Prosocial Behavior, *α* Cronbach’s Alpha, *ω* McDonald’s Omega, *ICC* Intra-class correlation coefficient, *GLB* Greatest Lower Bound

**Table 6:** Factor loadings and internal consistency of Model C

	Age 7–17			Age 7–12			Age 13–17		
Item	PB	IP	EP	PB	IP	EP	PB	IP	EP
skind	.60	0	0	.59	0	0	.59	0	0
helpout	.35	0	0	.31	0	0	.43	0	0
consid	.47	0	0	.47	0	0	.44	0	0
caring	.44	0	0	.43	0	0	.51	0	0
shares	.37	0	0	.22	0	0	.45	0	0
obeys	.65	0	0	.61	0	0	.67	0	0
friend	.38	0	0	.46	0	0	.39	0	0
popular	.50	0	0	.51	0	0	.43	0	0
clingy	0	.40	0	0	.35	0	0	.46	0
unhappy	0	.72	0	0	.70	0	0	.72	0
bullied	0	.64	0	0	.66	0	0	.52	0
worries	0	.63	0	0	.54	0	0	.56	0
somatic	0	.45	0	0	.38	0	0	.49	0
loner	0	.36	0	0	.40	0	0	.44	0
oldbest	0	.23	0	0	.22	0	0	.31	0
afraid	0	.57	0	0	.60	0	0	.53	0
fidgety	0	0	.43	0	0	.45	0	0	.43
restles	0	0	.48	0	0	.41	0	0	.50
tantrum	0	0	.40	0	0	.49	0	0	.44
distrac	0	0	.50	0	0	.52	0	0	.51
lies	0	0	.44	0	0	.40	0	0	.53
fights	0	0	.50	0	0	.50	0	0	.56
reflect	0	0	−.45	0	0	−.41	0	0	−.52
attends	0	0	−.58	0	0	−.53	0	0	−.58
steals	0	0	.51	0	0	.55	0	0	.60
α	.71	.72	.44	.69	.70	.41	.73	.72	.48
ω	.61	.60	.22	.58	.57	.25	.62	.61	.28
ICC	.59	.63	.39	.55	.62	.36	.62	.64	.41
GLB	.64	.73	.59	.69	.71	.51	.65	.73	.62

*PB* Prosocial Behavior, *IP* Internalizing Problems, *EP* Externalizing Problems, *α* Cronbach’s Alpha, *ω* McDonald’s Omega, *ICC* Intra-class correlation coefficient, *GLB* Greatest Lower Bound

**Table 7:** Factor loadings and internal consistency of Model D

	Age 7–17					Age 7–12					Age 13–17				
Item	ES	H	PP	BP	PB	ES	H	PP	BP	PB	ES	H	PP	BP	PB
somatic	.47	0	0	0	0	.39	0	0	0	0	.53	0	0	0	0
worries	.65	0	0	0	0	.56	0	0	0	0	.57	0	0	0	0
unhappy	.75	0	0	0	0	.74	0	0	0	0	.77	0	0	0	0
clingy	.40	0	0	0	0	.36	0	0	0	0	.47	0	0	0	0
afraid	.58	0	0	0	0	.62	0	0	0	0	.56	0	0	0	0
restles	0	.50	0	0	0	0	.43	0	0	0	0	.53	0	0	0
fidgety	0	.44	0	0	0	0	.46	0	0	0	0	.45	0	0	0
distrac	0	.51	0	0	0	0	.53	0	0	0	0	.53	0	0	0
reflect	0	−.46	0	0	0	0	−.41	0	0	0	0	−.54	0	0	0
attends	0	−.60	0	0	0	0	−.54	0	0	0	0	−.61	0	0	0
loner	0	0	.41	0	0	0	0	.41	0	0	0	0	.45	0	0
friend	0	0	−.26	0	0	0	0	−.29	0	0	0	0	−.24	0	0
popular	0	0	−.39	0	0	0	0	−.35	0	0	0	0	−.36	0	0
bullied	0	0	.65	0	0	0	0	.65	0	0	0	0	.53	0	0
oldbest	0	0	.20	0	0	0	0	.22	0	0	0	0	.27	0	0
tantrum	0	0	0	.38	0	0	0	0	.45	0	0	0	0	.43	0
obeys	0	0	0	−.53	0	0	0	0	−.44	0	0	0	0	−.58	0
fights	0	0	0	.49	0	0	0	0	.47	0	0	0	0	.57	0
lies	0	0	0	.43	0	0	0	0	.38	0	0	0	0	.53	0
steals	0	0	0	.49	0	0	0	0	.52	0	0	0	0	.60	0
consid	0	0	0	0	.53	0	0	0	0	.51	0	0	0	0	.47
shares	0	0	0	0	.39	0	0	0	0	.24	0	0	0	0	.48
caring	0	0	0	0	.48	0	0	0	0	.48	0	0	0	0	.55
kind	0	0	0	0	.68	0	0	0	0	.64	0	0	0	0	.65
helpout	0	0	0	0	.37	0	0	0	0	.31	0	0	0	0	.48
α	.70	.17	.18	.22	.62	.66	.16	.17	.23	.57	.71	.07	.04	.34	.65
ω	.62	.12	.05	.22	.52	.58	.15	.08	.25	.47	.61	.11	.04	.32	.55
ICC	.58	.14	.15	.25	.50	.57	.18	.15	.15	.42	.62	.11	.08	.26	.53
GLB	.67	.38	.29	.44	.54	.66	.37	.31	.38	.45	.71	.45	.27	.50	.57

*ES* Emotional Symptoms, *H* Hyperactivity, *PP* Peer Problems, *BP* Behavior Problems, *PB* Prosocial Behavior, *α* Cronbach’s Alpha, *ω* McDonald’s Omega, *ICC* Intra-class correlation coefficient, *GLB* Greatest Lower Bound

A summary of the goodness of fit indexes for the four models tested across age groups is presented in Table 8.

**Table 8:** Fit statistics for the four models

Fit Index/Age group	Model A			Model B			Model C			Model D		
	Age 7–17	Age 7–12	Age 13–17	Age 7–17	Age 7–12	Age 13–17	Age 7–17	Age 7–12	Age 13–17	Age 7–17	Age 7–12	Age 13–17
χ^2^	980.05	741.64	971.81	1091.72	806.52	1148.45	882.33	640.33	953.04	1025.34	773.28	1056.27
df	265	265	265	272	272	272	272	272	272	268	268	268
p	0	0	0	0	0	0	0	0	0	0	0	0
CFI	0.83	0.87	0.86	0.81	0.85	0.83	0.86	0.90	0.87	0.82	0.86	0.85
TLI	0.81	0.85	0.84	0.79	0.84	0.81	0.84	0.89	0.85	0.80	0.84	0.83
RMSEA	0.06	0.05	0.06	0.06	0.05	0.07	0.06	0.04	0.06	0.06	0.05	0.06
WRMR	1.67	1.46	1.67	1.77	1.52	1.81	1.59	1.35	1.65	1.712	1.49	1.74

χ^2^ Chi-square test, *CFI* Comparative Fit Index, *TLI* Tucker-Lewis Index, *RMSEA* Root Mean Square Error of Approximation, *WRMR* Weighted Root Mean Square

The confirmatory analysis was performed in the four versions of the questionnaire to be evaluated. First, the original five-factor model has mediocre fit (χ^2^*(df) =* 980.46 (265), CFI = .834, TLI = .812, RMSEA = .061, WRMR *=* 1.673) Although all the loadings are statistically significant, there are five items which loadings are equal or below a threshold of .4 (solitary, has good friend, better with adults than with children, tempers, often volunteers). The goodness of fit indexes remain insufficient in the three groups.

Second, model B shows a slight lessening in the goodness of fit measurements (χ^2^*(df)* = 1091.724. (272), CFI = .81, TLI = .79, RMSEA *=* .064, WRMR *=* 1.766). All the loadings are statistically significant with seven items with values are lesser or equal than .4 (nervous in new situations, solitary, has a good friend, generally liked, better with adults than with children, shares readily and often volunteers). There is not satisfactory goodness of fit in any of the age categories.

Third, Model C shows a tenuous improvement compared to the other models. Goodness of fit measurements improve (χ^2^ *(df)* = 882.328 (272), CFI *=* .86, TLI *=* .844, RMSEA *= .*055, WRMR *=* 1.588) but six items have loadings lesser or equal than .4 (often volunteers, shares readily, has good friend, nervous in new situations, solitary and better with adults than with children). A slight improvement in the goodness of fit indexes is noted in the category of 7 to 12 years old. Nonetheless, it remains insufficient.

Finally, a five-factor second order model shows no major improvement over the three models above (χ^2^ *(df)* = 1025.335 (268), CFI *=* .824, TLI *=* .803, RMSEA *= .*062, WRMR *=* 1.712). Once again, seven items are equal to or fall below the threshold of 0.4.

### Internal consistency

Cronbach’s alpha and McDonald’s omega show great variation among the subscales of the four models. First, the analysis performed in the five-factor original model reports low Cronbach’s alpha coefficients in each subscale (ranging from .173 to .7). Similarly, McDonald’s omega scores on each subscale range from .04 to .616. GLB values range from .291 to .669 and ICC ranges from .144 to .58. The peer subscale has the lowest omega coefficient and the second lowest Cronbach’s alpha besides having three of its five factors loading below .4 value. Same values of internal consistency are observed in Model D since it groups the same items in five first-order factors. There is little yet insufficient improvement of those coefficients in some subscales of the SDQ in the sample of children from 13 to 17 years old.

Second, model B presents higher reliability coefficients than the original version (α = .601, ω = .453, ICC = .565, GLB = .662; α = .335, ω = .23, ICC = .307, GLB = .531; and α = .621, ω = .524, ICC = .5, GLB = .542, for internalizing, conduct and prosocial subscales respectively). The internal consistency improves among children from 13 to 17 years old and worsens in children between 7 to 12 years old. Despite the improvement in the coefficients, the reliability of the scale is still questionable.

Third, model C shows higher reliability coefficients than models A, B, and D (α = .714, ω = .606, ICC = .6, GLB = .692; α=. 717, ω=. 604, ICC = .63, GLB = .687; and α=. 444, ω = .222, ICC = .385, GLB = .612, for prosocial, internalizing and externalizing subscales respectively). The externalizing subscale has the lowest reliability among the three subscales. Besides, internal consistency tenuously improve in the sample of children from 13 to 17 years old.

Globally, the questionnaire presents insufficient reliability (α = .625, ω = .433, ICC = .613, and GLB = .696).

### Measurement invariance

Finally, the psychometric equivalence or measurement invariance across age group and biological sex are presented in Table 9.

**Table 9:** Multi-group measurement invariance

Variable	CFI	RMSEA	ΔCFI	ΔRMSEA
Age				
Configural invariance	.819	.05	NA	NA
Metric invariance	.827	.048	.008	.002
Scalar invariance	.78	.053	.047	.005
Latent mean’s invariance	.759	.056	.021	.002
Sex				
Configural invariance	.8	.053	NA	NA
Metric invariance	.814	.05	.014	.003
Scalar invariance	.787	.053	.027	.003
Latent mean’s invariance	.769	.055	.019	.002

Measurement invariance analysis was performed only with the second version of the three-factor model (Model C) which presents the best validity and reliability results. First, regarding age, the sample is split into two groups: children from 7 to 12 years old, and children whose ages are between 13 and 17 years old. There is evidence of metric invariance (ΔCFI = .008; ΔRMSEA = .002), but not of scalar invariance (ΔCFI = .047; ΔRMSEA = 0.005), nor latent means invariance (ΔCFI = .021; ΔRMSEA = .002). As shown in Table 7, values across the biological sex of the respondent also reveal no psychometric equivalence between girls and boys. There is not metric invariance (ΔCFI = .014; ΔRMSEA = .003), nor scalar invariance (ΔCFI = .027; ΔRMSEA = .003), nor latent means invariance (ΔCFI = .019; ΔRMSEA = .002).

## Discussion

The Strengths and Difficulties Questionnaire is a widely used instrument to assess children’s behaviour. However, its validity and reliability in the Ecuadorian context have not been a subject of study.

Considering that there are several internal factor structures reported in other studies around the world, this paper aimed to find the internal structure that has the best psychometric properties. A sample of 1470 students from 9 educational institutions participated in this study. The idiomatic adaptation of the SDQ was made by a multidisciplinary group which made slight changes in the Spanish version.

The sample was randomly divided into two subsets in order to perform a factor analysis of the SDQ. On the one hand, the exploratory factor analysis would show whether the original five-factor structure can be found in the first subset of the data. This analysis revealed that more than five dimensions could be extracted from the SDQ, leading to consider other internal factor structures. On the other hand, four different internal factor structures were tested using CFA in the second subset. A combination of fit indices was used to assess the construct validity of the SDQ. The results of this analysis show questionable construct validity.

The SDQ internal structure is a matter of discussion. Initially, the items and subscales were elaborated based on contemporary classifications systems of child mental disorders [30]. The SDQ is considered by the literature to work as good as the Rutter questionnaires, but this paper shows that the interpretation of its scores must be made with caution. For instance, recent research [25] points out that different populations might show what is considered normal behaviour differs significantly across groups. Bird [45] suggests that certain words or questions might be differently understood by children in a non-western context. For instance, in Gaza [24], despite that the SDQ might be used as a screening measure across groups, there are indigenous constructs that might not be entirely captured by the 25 items of the questionnaire. Several researchers show questionable reliability and validity indexes in the conduct and peer problems subscale; the fact that there are only five questions that attempt to measure one construct might not adequately capture other more heterogeneous constructs that might be present in other cultures [25]. Other research suggests that bad psychometric properties might be an outcome of deficient reading abilities of children under 13 years old. Despite that in all the four models, the internal consistency is higher in the category of children from 13 to 17 years old and lower in the category of children from 7 to 12 years old, such improvement is tenous and insufficient. At the same time, the goodness of fit indices do not reveal better psychometric properties in this category.

In the Ecuadorian context, the factor loadings of four items (“Rather solitary, prefers to play alone”; “Has at least one good friend”; “Gets along better with adults than with other children”; “Often offers to help others (parents, teachers, other children)”) are equal or below .4 in all the models evaluated which show that these items might have a different meaning. Furthermore, two items (“Easily distracted, concentration wanders”; “Shares readily with other children, for example, toys, treats, pencils)”) also present weak loading in models B and C. When analyzing the item-total correlations the five items with the lowest coefficients are the ones with low factor loadings: “Gets along better with adults than with other children”; “Often offers to help others (parents, teachers, other children)”; “Has at least one good friend”; “Shares readily with other children, for example toys, treats, pencils”; and, “Helpful if someone is hurt, upset or feeling ill)”.

Model C revealed better psychometric properties than models A, B, and D. In model C, despite the RMSEA is below .08, both CFI and TLI fail to reach the threshold value of .9.

Assessment of the reliability of the SDQ reveals low coefficients of Cronbach’s Alpha, McDonald’s Omega, Intra-class correlation coefficient, and Greatest Lower Bound. Model C performs better out of the four models. However, the internal consistency coefficients for the prosocial behaviour and internalizing problems are barely acceptable, while the externalizing problems subscale reveals a lack of reliability.

Invariance of the instrument was tested using model C since it has, relatively, the best validity and reliability indexes. There is no evidence of scalar and latent means invariance across age groups, only metric invariance. Regarding sex, there is no evidence of metric, scalar and latent means invariance. The invariance of an instrument means that a construct has psychometric equivalence across groups. Consequently, measurement invariance analysis is recommended before making comparisons. The analysis performed in the SDQ does not back this claim. Therefore, comparisons between boys and girls should not be performed. Furthermore, the analysis reveals that there is indeed a difference between children that are below 13 years old and those who are older than 13, but psychometric properties remain poor when the data is stratified suggesting that the poor psychometric properties might not only be a result of insufficient reading abilities as suggested in other research.

## Conclusions

Four models were evaluated showing that the second version of the three-factor model used in several investigations [18, 19, 22] presents better psychometric properties than the other three versions. The original five-factor structure model seems to be inappropriate for its use in the Ecuadorian context since it shows mediocre goodness of fit indexes and internal consistency. Among the three studied models, Model C has the best yet insufficient validity and reliability coefficients.

More research is necessary that might lead to change in the structure of the questions or fully understand the hidden constructs that might be present among children and adolescents of Biblián, Ecuador.

The prosocial behaviour and the internalizing problems subscale reported in Model C has barely acceptable internal consistency. Consequently, only these subscales of the SDQ should be used but interpreted with caution when screening for psychopathological symptoms and jointly with other scales.

## Data Availability

The de-identified datasets used and/or analysed during the current study are available from the corresponding author on reasonable request.

## Abbreviations

CFA: Confirmatory Factor Analysis
CFI: Comparative Fit Index
EFA: Exploratory Factor Analysis
GLB: Greatest Lower Bound
ICC: Intra-class Correlation Coefficient
RMSEA: Root-Mean-Square Error of Approximation
SDQ: Strengths and Difficulties Questionnaire
TLI: Tucker-Lewis Index
WRMR: Weighted Root-Mean-square Residual

## References

[1] Polanczyk GV, Salum GA, Sugaya LS, Caye A, Rohde LA (2015). Annual research review: a meta-analysis of the worldwide prevalence of mental disorders in children and adolescents. J Child Psychol Psychiatry Allied Discip.

[2] Goodman R (1999). The extended version of the strengths and difficulties questionnaire as a guide to child psychiatric caseness and consequent burden. J Child Psychol Psychiatry Allied Discip.

[3] Goodman R (1994). A modified version of the Rutter parent questionnaire including extra items on Children’s strengths: a research note. J Child Psychol Psychiatry.

[4] Goodman R (2001). Psychometric properties of the strengths and difficulties questionnaire. J Am Acad Child Adolesc Psychiatry.

[5] Goodman R, Meltzer H, Bailey V (2003). The strengths and difficulties questionnaire: a pilot study on the validity of the self-report version. Int Rev Psychiatry.

[6] Muris P, Meesters C, Eijkelenboom A, Vincken M (2004). The self-report version of the strengths and difficulties questionnaire: its psychometric properties in 8- to 13-year-old non-clinical children. Br J Clin Psychol.

[7] Curvis W, McNulty S, Qualter P. The validation of the self-report strengths and difficulties questionnaire for use by 6- to 10-year-old children in the UK. Br J Clin Psychol. 2014.10.1111/bjc.1202524588764

[8] Patalay P, Hayes D, Wolpert M (2018). Assessing the readability of the self-reported Strengths and Difficulties Questionnaire. BJPsych Open.

[9] Cucchiaro G, Dalgalarrondo P (2007). Mental health and quality of life in pre- and early adolescents: a school-based study in two contrasting urban areas. Rev Bras Psiquiatr.

[10] Cury Camilo Ramos, Golfeto José Hércules (2003). Strengths and difficulties questionnaire (SDQ): a study of school children in Ribeirão Preto. Revista Brasileira de Psiquiatria.

[11] Goodman R, Renfrew D, Mullick M (2000). Predicting type of psychiatric disorder from strengths and difficulties questionnaire (SDQ) scores in child mental health clinics in London and Dhaka. Eur Child Adolesc Psychiatry.

[12] Goodman A, Goodman R (2009). Strengths and difficulties questionnaire as a dimensional measure of child mental health. J Am Acad Child Adolesc Psychiatry.

[13] Fletcher J, Tannock R, Bishop DVM (2001). Utility of brief teacher rating scales to identify children with educational problems: experience with an Australian sample. Aust J Psychol.

[14] Hawes DJ, Dadds MR (2004). Australian data and psychometric properties of the strengths and difficulties questionnaire. Aust N Z J Psychiatry.

[15] Mellor D, Stokes M (2007). The factor structure of the strengths and difficulties questionnaire. Eur J Psychol Assess.

[16] Mullick MSI, Goodman R (2001). Questionnaire screening for mental health problems in Bangladeshi children: a preliminary study. Soc Psychiatry Psychiatr Epidemiol.

[17] Dickey WC, Blumberg SJ (2004). Revisiting the factor structure of the strengths and difficulties questionnaire: United States, 2001. J Am Acad Child Adolesc Psychiatry.

[18] Koskelainen M, Sourander A, Vauras M (2001). Self-reported strengths and difficulties in a community sample of Finnish adolescents. Eur Child Adolesc Psychiatry.

[19] Van Leeuwen K, Meerschaert T, Bosmans G, De Medts L, Braet C (2006). The strengths and difficulties questionnaire in a community sample of young children in flanders. Eur J Psychol Assess.

[20] Ortuño-Sierra J, Fonseca-Pedrero E, Paino M, Sastre I, Riba S, Muñiz J (2015). Screening mental health problems during adolescence: psychometric properties of the Spanish version of the strengths and difficulties questionnaire. J Adolesc.

[21] Ortuño-Sierra J, Chocarro E, Fonseca-Pedrero E, Riba SSI, Muñiz J (2015). The assessment of emotional and Behavioural problems: internal structure of the strengths and difficulties questionnaire. Int J Clin Health Psychol.

[22] Di Riso D, Salcuni S, Chessa D, Raudino A, Lis A, Altoè G (2010). The strengths and difficulties questionnaire (SDQ). Early evidence of its reliability and validity in a community sample of Italian children. Personal Individ Differ.

[23] Giannakopoulos G, Tzavara C, Dimitrakaki C, Kolaitis G, Rotsika V, Tountas Y (2009). The factor structure of the strengths and difficulties questionnaire (SDQ) in Greek adolescents. Ann General Psychiatry.

[24] Thabet AA, Stretch D, Vostanis P (2000). Child mental health problems in Arab children: application of the strengths and difficulties questionnaire. Int J Soc Psychiatry.

[25] Du Y, Kou J, Coghill D (2008). The validity, reliability and normative scores of the parent, teacher and self report versions of the strengths and difficulties questionnaire in China. Child Adolesc Psychiatry Ment Health.

[26] Ortuño-Sierra J, Fonseca-Pedrero E, Aritio-Solana R, Velasco AM, de Luis EC, Schumann G (2015). New evidence of factor structure and measurement invariance of the SDQ across five European nations. Eur Child Adolesc Psychiatry.

[27] Bøe T, Hysing M, Skogen JC, Breivik K (2016). The Strengths and Difficulties Questionnaire (SDQ): Factor structure and gender equivalence in Norwegian adolescents. PLoS One.

[28] Smedje H, Broman JE, Hetta J, von Knorring AL (1999). Psychometric properties of a Swedish version of the ‘strengths and difficulties questionnaire’. Eur Child Adolesc Psychiatry.

[29] Woerner W, Fleitlich-Bilyk B, Martinussen R, Fletcher J, Cucchiaro G, Dalgalarrondo P (2004). The strengths and difficulties questionnaire overseas: evaluations and applications of the SDQ beyond Europe. Eur Child Adolesc Psychiatry, Suppl.

[30] Goodman A, Lamping DL, Ploubidis GB (2010). When to use broader internalising and externalising subscales instead of the hypothesised five subscales on the strengths and difficulties questionnaire (SDQ): data from british parents, teachers and children. J Abnorm Child Psychol.

[31] Cronbach LJ (1951). Coefficient alpha and the internal structure of tests. Psychometrika..

[32] McDonald RP. Test theory: A unified treatment. Test theory A unified treatment. 1999;:485.

[33] Ten Berge JMF, Sočan G (2004). The greatest lower bound to the reliability of a test and the hypothesis of unidimensionality. Psychometrika..

[34] Kaiser HF (1960). The application of electronic computers to factor analysis. Educ Psychol Meas.

[35] Beauducel A, Herzberg PY (2006). On the performance of maximum likelihood versus means and variance adjusted weighted least squares estimation in CFA. Struct Equ Model.

[36] Flora DB, Curran PJ (2004). An empirical evaluation of alternative methods of estimation for confirmatory factor analysis with ordinal data. Psychol Methods.

[37] Lei PW (2009). Evaluating estimation methods for ordinal data in structural equation modeling. Qual Quant.

[38] Li C-H (2014). The performance of MLR, USLMV, and WLSMV estimation in structural regression models with ordinal variables.

[39] Bentler PM (1990). Comparative fit indexes in structural models. Psychol Bull.

[40] Browne MW, Cudeck R (1992). Alternative ways of assessing model fit. Sociol Methods Res.

[41] Hu LT, Bentler PM (1999). Cutoff criteria for fit indexes in covariance structure analysis: conventional criteria versus new alternatives. Struct Equ Model.

[42] Yu CY. Evaluating cutoff criteria of model fit indices for latent variable models with binary and continous outcomes. 2002. doi:10.1.1.310.3956.

[43] Rosseel Y (2012). lavaan: An R Package for Structural Equation Modeling. J Stat Softw.

[44] Kaiser HF, Rice J (1974). Little jiffy, Mark Iv. Educ Psychol Meas.

[45] Bird HR (1996). Epidemiology of childhood disorders in a cross-cultural context. J Child Psychol Psychiatry Allied Discip.

